RETRACTED

# Prediction and Risk Assessment Models for Subarachnoid Hemorrhage: A Systematic Review on Case Studies

**DOI:** 10.1155/2022/5416726

**Published:** 2022-01-27

**Authors:** Jewel Sengupta, Robertas Alzbutas

**Affiliations:** Kaunas University of Technology, K. Donelaičio g. 73, Kaunas 44249, Lithuania

## Abstract

Subarachnoid hemorrhage (SAH) is one of the major health issues known to society and has a higher mortality rate. The clinical factors with computed tomography (CT), magnetic resonance image (MRI), and electroencephalography (EEG) data were used to evaluate the performance of the developed method. In this paper, various methods such as statistical analysis, logistic regression, machine learning, and deep learning methods were used in the prediction and detection of SAH which are reviewed. The advantages and limitations of SAH prediction and risk assessment methods are also being reviewed. Most of the existing methods were evaluated on the collected dataset for the SAH prediction. In some researches, deep learning methods were applied, which resulted in higher performance in the prediction process. EEG data were applied in the existing methods for the prediction process, and these methods demonstrated higher performance. However, the existing methods have the limitations of overfitting problems, imbalance data problems, and lower efficiency in feature analysis. The artificial neural network (ANN) and support vector machine (SVM) methods have been applied for the prediction process, and considerably higher performance is achieved by using this method.

## 1. Introduction

Acute brain injuries are very serious health issues that require early care for effective treatment of the patient. Advancements in neurosurgical and critical care techniques help to increase the survival rate [1, 2]. The functional outcomes of an individual suffering from such injuries are very fatal and lead to secondary complications such as seizures, inflammation, and brain swelling, most of which are potentially amenable if proper therapy is used for treatment [3, 4]. Subarachnoid aneurysmal hemorrhage (SAH) is a brain-related injury and is considered a major health issue among the many existing ones in society. The SAH occurs 9.1 per 100000 people annually worldwide, and studies from Japan and Finland have 22.7 and 19.7, respectively [5]. Detection, prevention, and the clinical management of these secondary complications are large burden for the health care centers dealing with SAH patients [6, 7]. Among aneurysmal SAH (aSAH), the delayed cerebral ischemia (DCI) is the major cause of mortality [8, 9]. For suspected SAH patients, computed tomography (CT) is the preferred method for imaging due to its wide availability and high sensitivity [10, 11]. Magnetic resonance imaging (MRI) is considered equally or more sensitive than CT for acute or subacute SAH detection [12]. Electroencephalography (EEG) signal provides information about the cortical activity in the brain [13]. Fast activity depression and rhythms slowing changes EEG signals when insufficient cortical perfusion compromised the neuronal function [14]. EEG signals are applied in some researches, for the detection of DCI at an early stage [15–17].

RETRACTED

Early diagnosis and treatment of SAH patients are important to ensure optimal cerebral blood flow and will also potentially improve the long-term outcome of patient's health [18, 19]. Some researchers are considering that changes in heart rate variability (HRV) with clinical events provide relevant features for prediction [20, 21]. Large cerebral artery vasospasm is associated with the risk of DCI and SAH, but vasospasm cannot be considered as a strong factor for predicting DCI [22, 23]. The aSAH patient's clinical features such as heart rate, blood pressures, intracranial pressures (ICP) [24], glucose and sodium values [25], and drainage volumes of cerebrospinal fluid (CSF) [26] were monitored and not applied for the prediction of SAH and symptoms of SAH. Reliable prediction of aSAH is based on various factors that act as a support system for resource allocation and treatment decisions. Clinical scoring systems and radiography help in the estimation of disease severity, and predictive value is limited in devising treatment strategies [27, 28]. Machine learning and deep learning methods were applied for the prediction of SAH and DCI for the effective treatment of the patients [29, 30]. In this paper, prediction models such as statistical analysis, machine learning, and deep learning models that are used for SAH prediction are reviewed along with each model's advantages and limitations.

The organization of this paper is given as follows: a review of various prediction models of SAH with statistical analysis, logistic regression, machine learning, and deep learning models are reviewed in Section 2, and comparative analysis of various models in SAH is given in Section 3, and a conclusion is given in Section 4.

## 2. Review of SAH Prediction Models

The SAH prediction model involves the application of machine learning or statistical method applied in clinical factors, CT, MRI, and EEG data. In this review, the statistical method, machine learning, and deep learning method applied for the clinical factors for SAH prediction were reviewed. Generally, prediction of SAH involves in dataset collection and application of the classifier to assess the risk or predict the SAH. Some of the researches involve in applying the medical images like CT, MRI, EEG signal, and clinical factors for the SAH prediction. Statistical analysis and regression were also used for the risk assessment in the SAH prediction. Some of the standard machine learning techniques such as SVM, RF, and ANN were applied for the prediction of SAH. Machine learning methods involve in learning the features with its label in training process. For instances, random forest method involves in development of the tree based on the given features in training and in testing; test data is applied in the tree structure to perform classification. Deep learning method is subpart of machine learning techniques that performs unsupervised classifier based on deep feature learning. Deep learning method like CNN-based model learns the features in the neurons without its label in the training process. The overview of the model is shown in Figure 1.

RETRACTED

### 2.1. Prediction Models

Various prediction models that were based on machine learning methods were applied for the early detection of SAH.

Steen et al. [31] carried out the statistical analysis based on the various clinical factors related to the patient. The Fisher model is used to evaluate the performance of the statistical model, and this shows statistical model has considerable efficiency in the analysis. The statistical method has lower efficiency in the feature analysis. Nassar et al. [32] applied statistical methods for the detection and prediction of the SAH. The Fisher and Monte Carlo method was used to evaluate the performance of the model. The EEG and CT data of 46 patients were used to evaluate the performance of the developed model. The feature analysis and feature relation analysis are not efficient in the model. The statistical methods consider the features in linear relation with output factor, and the model does not learn from the input data. Zeiler et al. [33] applied statistical analysis based on the Full Outline of UnResponsiveness (FOUR) measure for prediction of SAH. The collected data was used to evaluate the performance of the developed method. The evaluation shows that the developed method has considerable performance. The developed method has lower efficiency in feature analysis and feature relation analysis. Malinova et al. [34] applied statistical analysis in the CT images to predict the SAH. The CT perfusion data were used to evaluate the performance of the developed statistical model. The developed model has considerable performance in the prediction process based on CT perfusion features. The developed method has lower efficiency in the feature analysis and feature relation analysis.

RETRACTED

Kanazawa et al. [35] applied the Synapse Vincent software program for the prediction of SAH based on CT images. The texture features of CT and features such as mean CT value, kurtosis, and skewness were used in this prediction. The developed method showed considerable performance in the prediction of SAH. The texture features of the CT were not effectively detected in the model and lower performance in feature analysis. Park et al. [36] applied a statistical method for the prediction of SAH based on the clinical features of the patient data. The dataset of 418 patients was used to evaluate the performance of the model. The model achieved considerable performance in the prediction process of SAH. The feature analysis and feature relation analysis of clinical factors were not efficiently implemented in the model. Yan et al. [37] applied a multivariable logistic regression model with various clinical features for the prediction of SAH. The least absolute shrinkage and selection operator (LASSO) was used to select the predictive risk factors for patients with aSAH. The selection operator regression and least absolute shrinkage were applied to optimize the factor selection for the poor recovery risk model. The overfitting problem occurred in the model that affected the performance of the developed model.

Fang et al. [38] applied a statistical method for the prediction of SAH based on the modified Fisher scale. The collected data were used to evaluate the performance of the developed method in prediction. The analysis shows that the developed method has considerable performance in the analysis. Liu et al. [39] applied multivariate logistic regression for the prediction of SAH and analyzed independent risk factors. The model has considerable performance in the prediction process. The feature analysis and the feature relation analysis based on clinical factors are not efficiently implemented in the model. Lublinsky et al. [40] applied the logistic regression method for the prediction of SAH. The model has considerable performance in the prediction of SAH in the analysis. The logistic regression model is not stable and has lower efficiency in the prediction of SAH. Geraghty et al. [41] applied the logistic regression method for the prediction of the SAH in the patient data. The clinical factors were applied for the prediction of SAH in the developed method. The logistic regression has unstable performance, and overfitting problem had occurred in the prediction process.

### 2.2. Prediction Model Based on Machine Learning Techniques

Machine learning techniques demonstrate efficient performance in prediction, detection, and classification processes. The machine learning models were applied in the CT, MRI, and EEG data for the prediction of SAH.

RETRACTED

Rau et al. [42] applied the Classification And Regression Tree (CART) method for the prediction of SAH based on the Gini Index. The dataset with 545 patient data was used to evaluate the performance of the CART method. The CART method has considerable performance in the prediction process. The decision tree model is unstable and inefficient in the prediction process of SAH. Malik et al. [43] proposed a knowledge graph model for concept extraction, individual and relational feature analysis, and prediction process. Ensemble learning method based on skip-gram technique was applied to handle structured and unstructured data of patient records. The knowledge graph method showed higher performance in the feature analysis and prediction process of SAH. The developed model had lower efficiency due to an imbalance dataset and overfitting problem in the analysis. Kim et al. [44] applied convolutional neural network (CNN) for digital subtracting angiography. The collected dataset was applied to evaluate the performance of CNN in risk assessment. The developed model showed considerable performance in the prediction process. The overfitting problem in the CNN model affects the performance of the model.

Chen et al. [45] applied machine learning techniques in IoT for the diagnosis of a human brain hemorrhage. The feedforward neural network and support vector machine methods are applied for the CT dataset. The feedforward neural network achieved higher performance in the detection method. The support vector machine had lower efficiency in the detection method due to the data imbalance problem. Liu et al. [46] applied the SVM method with univariate and multivariate analysis for the prediction of hemorrhage based on CT data of patients. The collected data was used to evaluate the performance of the developed method. The analysis showed that the developed method has higher performance in the prediction of hemorrhage. The SVM method is lesser efficient due to the imbalance dataset. Govindarajan et al. [47] applied machine learning methods such as support vector machine, random forest, artificial neural network (ANN), boosting, and bagging for the prediction process. The artificial neural network with the stochastic gradient method achieved higher performance in the analysis. The developed method has an overfitting problem and lower efficiency in the imbalance dataset.

Zhu et al. [48] applied feed-forwarded ANN, SVM, and random forest with clinical and morphological features in the prediction model. The analysis of the prediction model's outcome shows that machine learning models have higher performance than statistical analysis. The ANN model has lower efficiency in the feature selection process for the prediction of hemorrhage. Cho et al. [49] presented a cascade deep learning method using two CNN models and dual fully convolutional networks. The CNN method is applied for five types of hemorrhages in the CT images. The CNN method had the overfitting problem that affected the performance of the method. Shahzad et al. [50] applied a deep learning model for the prediction of SAH in CT images. The deep learning methods with ensemble learning technique were applied to analyze the performance of the prediction. The deep learning method showed higher performance in the prediction process.

RETRACTED

Abujaber et al. [51] applied ANN and SVM method with clinical factors on CT images for the prediction. The ANN and SVM provide higher performance in the prediction process, and the optimal accuracy in the prediction is achieved by using SVM, but it proves to be less efficient while dealing with an imbalance dataset. Ginat [52] applied a deep learning method for the analysis of hemorrhage in CT images. The collected data was used to evaluate the performance of the developed model in prediction. Hong et al. [53] applied three machine learning techniques that are SVM, Naïve Bayes, and random forest for the detection of hemorrhagic brain. ReliefF feature selection method was applied to select the relevant features. The random forest achieved higher performance compared to other methods. Random forest is inefficient when a number of a tree is a high and overfitting problem when a number of trees are less.

Barros et al. [54] applied CNN for the detection and prediction of SAH in the noncontrast CT images. The collected data were used to evaluate the performance of the SAH prediction performance. The developed model showed higher performance in the segmentation and prediction. The CNN has an overfitting problem that affects the performance of the prediction method. Nawabi et al. [55] applied random forest with filter and texture-derived features for the prediction process. The developed method with the selected features achieved higher performance in the analysis.

Some methods follow the random forest method for the prediction process but the random forest method has the limitation of inefficient and overfitting in the training.

Claassen et al. [1] developed an Ensemble RF Algorithm for analyzing big data. As the dataset is imbalanced due to the missing features of business data and many more, reasons were noticed. Thus, the classification algorithms such as SVM and logistic regression algorithm faced difficulty to model the insurance business data. The developed model exploited a heuristic bootstrap sampling technique that combined the ensemble learning model for large-scale insurance business data. The developed model introduced an ensemble approach that performs computation tasks and optimized memory cache using spark mechanism. The ensemble approach combined the bootstrap sampling process that reduced the learning process and showed better reference for remaining imbalanced data mining algorithms. The developed ensemble approach has analyzed the big data and was applied for IoT, mobile Internet, and finance things. However, the developed model further works including exploration of proposed algorithm with distinct big data analytics such as combining with deep learning model improves the prediction accuracy based on big data.

RETRACTED

Fang et al. [4] utilized a RF approach for modelling the behavior for travel mode choice. The decision tree (DT) decorrelates in ensemble through randomization leading to improvement to forecast which reduces the variances. These were averaged over the trees, and the RF usefulness to travel mode choice behavior largely remained as unexplored. The developed model introduced a robustly approaching RF model that analyzed for travelling mode choices which examined the capability during model prediction and interpreted the model ability. The results obtained by the developed model showed that the RF model performed better measures significantly better with travel model choice prediction for obtaining accuracy better and with computation cost of less. Also, the developed model estimated that the explanatory variables showed relatively importance better and was related for mode choices. There are many benefits based on the machine learning behavioral interpretation which showed difficulty because of the complexity in the number of parameters of the system. The machine learning models performed research and rapidly showed intersection of statistical analysis, and information science discovered the complex patterns present on the datasets. The emphasis on theoretical and application investigation with respect to the present dataset showed improvement based on analytical techniques. These machine learning techniques were utilized in order to perform relevant, statistical, and probability theory for analyzing the econometric data which were still to be analyzed for travel behavior analysis. The random forest architecture is shown in Figure 2.

Chimmula and Zhang [56] developed long-short-term memory (LSTM) networks for time series forecasting for COVID-19 data belonging to Canada. The public dataset utilized was acquired at John Hopkins university from Canadian health authority. The developed model performed forecasting model for the COVID data using deep learning model. The key features were utilized for performing the trend prediction and also to find out the possible stopping time from that of the existing COVID data worldwide. The developed LSTM model predicted the ending point for the outbreak data and modeled the pandemic with respect to the people who were travelling. The results showed that the developed model obtained fruitful results as the current trails on vaccines were achieved.

RETRACTED

Kim and Cho [57] performed prediction of residential energy consumption based on the CNN-LSTM models. The electricity is generated by the power plant and is simultaneously consumed based on the stable power supply. The CNN-LSTM extracted the temporal and spatial features for predicting the energy consumption at the housing. The results obtained from the experiment have showed that the CNN-LSTM combined with CNN extracted the features related to energy which were complex in nature. From the CNN layer, the features extracted affected the energy consumption, and LSTM model modeled the temporal information. The information from the irregular trends were extracted from the time series components. The proposed CNN-LSTM model achieved prediction of performance with respect to electric energy which showed difficulty previously. The smallest value is recorded by evaluating the root mean square error which showed better values when compared with the conventional forecasting techniques from the dataset showed household power consumption individually. The model reflected large evaluation measures on the basis of trial and error method determined hyperparameters optimally. An automated searching found the best hyperparameters using genetic algorithm during the process. The developed model still required lots of houses for validating the model for evaluating the collected energy and the consumed energy data.

Park et al. [58] developed a LSTM-based battery for Remaining Useful Life (RUL) prediction with the help multichannel charging profiles. The developed model estimated RUL with the presence of capacity regeneration phenomenon that considered a multiple measured data from a battery managing system. The parameters such as current, temperature, and voltage were considered for charging the whole pattern profiles that varied with respect to ages. The existing LSTM traditional methods performed prediction that matched the output and input layer with respect to one after the other structure. The many to one structure showed flexibility with respect to distinct input types which reduced substantially the parameters that gave better process of generalization. The multichannel (MC) profiles were charged and exploited with respect to current, temperature, and voltage that were necessary for RUL prediction accurate. The developed MC-LSTM model showed better significance with respect to the baseline of the EoL leading the batteries to utilized better without declaring premature till the end of use.

RETRACTED

Shahid et al. [59] performed classification using deep learning models such as gated recurrent unit (GRU), bidirectional long-short-term memory (Bi-LSTM), and LSTM models. The developed model set up a strategic plan for developing a public health system in order to avoid the death and managing the patients. The dataset is comprised of 3 features that included data related to recovered cases, confirmed cases, and also deaths. The unscaled data slowed the process of convergence, and thus, min-max scalar was utilized for the preprocessing which subtracted the original value with the smallest feature value and divided the feature range. The range is known as the difference among the maximum feature value to the minimum feature value at original point. The min-max scalar reserved the original shape obtained from the data distributions. The forecasting model is comprised of autoregressive integrated moving average (ARIMA), support vector regression (SVR), long-shot-term memory (LSTM), and bidirectional long-short-term memory (Bi-LSTM) which assessed the time series prediction. The time series models predicted confirmed cases, recoveries, and also, deaths based on the time. Thus, by the result analysis, 10 major countries that were affected by COVID were determined. This concluded that an appropriate predictor Bi-LSTM model predicted data and enhanced based on the sequential data and predicted the accuracy for the datasets which required a suitable planning for managing it better.

Fu et al. [60] developed a CNN model using MRI images that performed segmentation. The developed DL model contained voxel wise label which was used for prediction and a correction network. The network consisted of 2 subnetworks that included dense blocks which consisted of 12 densely connections. The subnetworks were able to learn for overcoming the erroneous classification problem based on the previous network considering the original and input images which generated soft max probability based on the subnetwork previously. Each of the subnetworks was trained by parameters independently by using piece wise training. The developed model was used for presegmenting the 3D MRIs which were important for correcting manually for training the datasets and also preparing it. This expedites greatly the process of manual contouring which potentially faced the problem of dataset in medical image deep learning approach.

RETRACTED

Zou et al. [61] developed a 3D CNN model which performed an automated diagnosis of hyperactivity disorder based on the structural and functional MRI. The public dataset was available as a large neuroimaging dataset used for the process of training. The deep learning model was automatically diagnosed the disorder of psychiatric disorders which showed feasibility. The developed model utilized deep learning approach that performed ADHD for classification through 3D CNN applied to MRI. The deep neural network (DNN) model was utilized with distinct parameters that were large in number which acquired those data which was limited with discriminated features obtained from raw data. Thus, overfitting problem was overcome by using 3D CNN model that trained various methods. The 3D CNN model took it as an advantage of those intrinsic features which showed partial connectivity, pooled the architectures, and shared the weights. The developed model designed the various number of layers and mapped the features which avoided overfitting problem but retained sufficient network capacity which solved the ADHD classification problems. Data augmentation was performed for the drop out layer and contained the weights in the network. The 3D CNN model was trained and yielded better results in terms of accuracy. The developed model considered 3D low-level features extracted from structural and functional MRI data. The data augmentation was performed through dropout technique which was connected with layers containing weights in the network. The results showed that the proposed 3D CNN was trained and thus yielded better results compared to existing models. The developed model was investigated; ADHD testing dataset showed superiority in the performances compared to other approaches for few training samples. The architecture of DNN is shown in Figure 3.

Iqbal et al. [62] performed segmentation of brain tumor using multispectral MRI based on CNN. The CNN model set up various techniques for providing results better compared with the nondeep learning techniques which segmented the brain tumor parts. The developed model used CNN for segmenting the brain tumor regions using the MRIs. The BRATS dataset was used for performing the segmentation that showed challenge when composed with images that showed different modalities. The extended version of the model solved the segmentation problem due to the multiple layers. The network architecture has multiple layers sequentially connected to feed the CNN feature maps at their high level. The developed model has a very small structure, less memory, and fast for demanding. The SE blocks were explored at distinct levels and explored that the type of weighting strategy was better and showed good results for combined classifier.

RETRACTED

Mortazi et al. [63] developed a CardiacNET which performed segmentation of proximal pulmonary veins and left atrium from MRI using CNN model. The developed model addressed the need of unmet clinical-based technologies using deep learning-based segmentation technique for separating LA and PPVs which obtained classification accuracy at high rate and improved the efficiency. The developed approach utilized a multiview CNN model which performed fusion by using an adaptive strategy that allowed loss function operating faster and accurate improving its convergence using the optimization approach known as back propagation algorithm. The network model will be trained from the beginning that has more than 60K 2D MRI slices of images, and also, STACOM 2013 was utilized for performing cardiac segmentation which showed difficulty by the benchmark dataset. The novel method is going to be evaluated, tested, and will be validated with more distinct datasets that consisted of various cohorts operated at distinct imaging resolution images with noises at high levels across the scanner vendors distinctly. The framework was extended to 4D which analyzed the cardiac images that extended the possible parsing technique. However, the exploration of 3D cardiac MRI required complete training on the basis of the multiple GPUs that would overcome the segmentation problem by CNN.

The feature learning methods with random forest [64–68] methods can be applied to improve the prediction performance. In deep learning methods, LSTM [56–59, 69] can be applied for the clinical feature analysis, and CNN models [60–63, 70] can be applied for the CT and MRI images. The feature learning methods like principal component analysis and *k*-mean methods help to improve the performance of models. The evolutionary optimization methods such as Ant Colony Optimization (ACO) and FireFly optimization were applied to improve the learning performance of classifier model.

### 2.3. Datasets

The intracranial hemorrhage dataset (https://www.kaggle.com/c/rsna-intracranial-hemorrhage-detection) consists of CT scans of 25,000 exams from 60 subjects for classification of hemorrhage [71–75]. The sample images of RSNA intracranial hemorrhage is shown in Figure 4. The study [34] collected 128 CT images from the Siemens Healthcare Sector, Forchheim, Germany. The study [35] collected CT images of 40 patients from Keio University Hospital between 2015 and August 2018. The study [36] collected 418 CT images from hospitals to analyze the performance. The study [37] collected 1577 patients from the Department of Neurosurgery of five Chinese hospitals located in China from January 2017 to December 2018.

RETRACTED

## 3. Comparative Analysis

Subarachnoid hemorrhage (SAH) is a major health issue that has a higher mortality rate, and it leads to functional disability of the person suffering from it. Some researchers involved in applying machine learning and deep learning techniques for the prediction of SAH. Recent, notable researches that were used in the prediction and monitoring of SAH are reviewed along with the advantages and limitations of these researched methods in Table 1.

### 3.1. Challenges in Prediction of SAH

From the reviews of various methods in the prediction of SAH, there are some of the common limitations in the existing methods of SAH prediction.

SVM methods applied in the existing SAH prediction have the limitation of the model biased to class with high instances. SVM method learns the instances in the vector, and hyperplane models classify the data instances bias to the class.

Random forest method in SAH prediction has overfitting problem when number of tree is low and instable performance when number of tree is high in the model development.

CNN model generates the weight values for the input features and performs the classification based on convolution and pooling data. The generation of more feature values involves in creating the overfitting of the neural network.

## 4. Conclusion

SAH is considered one of the major health issues and has a higher mortality rate among SAH patients. Prediction of SAH and risk assessment helps to effectively treat the patient and considered as a decision model. SAH prediction and risk assessment involve the analysis of clinical factors, CT, MRI, and EEG data. Existing methods involve applying the statistical method, logistic regression, machine learning, and deep learning methods. In this paper, a review of various prediction models, used in SAH prediction, were carried out. The advantages and limitations of the prediction models were analyzed comparatively. Some researches involved the application of EEG data that gave more accurate results in the SAH prediction process. The analysis shows that machine learning methods are more efficient in their performance compared to the statistical and logistic regression methods. Random forest, ANN, and SVM show considerable performance in the prediction of SAH. The random forest consists of two limitations: first is it has lower efficiency when some trees are high, and second is the occurrence of the overfitting problem when the number of trees is less. SVM and ANN methods are less efficient in handling imbalanced datasets. The deep learning method of CNN has higher efficiency in the SAH prediction but has the limitation of overfitting problem. The future research works regarding SAH prediction will involve the application of the LSTM model in the analysis of clinical factors and application of CNN in CT, MRI, and EEG data of SAH patients.

RETRACTED

## Figures and Tables

**Figure 1:** The overview of the SAH prediction model.

**Figure 2:** Architecture of random forest.

**Figure 3:** Architecture of deep neural network (DNN).

**Figure 4:** Sample images of RSNA intracranial hemorrhage dataset.

**Table 1:** Comparative analysis of the prediction methods used for detection of SAH.

Method	Dataset	Advantages	Limitations
Applied random kernels to extract the features from physiological time series features [76]. Classifiers such as kernel SVM and partial least square were applied for prediction. The model was evaluated on the 488 consecutive data from a tertiary care hospital.	Dataset is collected from Columbia University Medical Center.	The evaluation shows that random kernel and kernel SVM has considerable performance in the prediction.	The feature relations are not effectively analyzed due to applied kernel function and SVM has lower performance in handling imbalance dataset. SVM requires more data instances to develop the optimal hyperplane.
*K*-nearest neighbor (KNN) was applied to impute the missing data [77]. Classifiers such as deep learning, gradient boosting machine, gradient boosting machine, and generalized linear modeling were used. The method was evaluated in 300 patient datasets.	Dataset is collected from the National Institute of Health Stroke Scale.	The analysis shows that the developed model has considerable performance in the prediction. The model has considerable performance in a large dataset.	KNN method computes the distance between the new data instance and the existing data instance. The distance calculation for high dimensions creates the overfitting problem in training. The overfitting problem has affected the performance of the model.
Deep learning and Grapcut-based segmentation were carried out for segmentation of SAH [78]. The deep learning method is applied for feature extraction, and the softmax method is applied for classification. The Benchmark dataset was used to evaluate the performance.	Physionet benchmark dataset	The deep learning and Grabcut method have higher efficiency in the segmentation. The model has higher performance in the benchmark dataset.	The convolution and upsampling of data in the deep learning model creates an overfitting problem. The model has an overfitting problem that affects the performance. The model has lower efficiency in imbalance dataset due to model requires more data instance for the class to train.
Correlation with the clinical and radiologic findings are analyzed in the model [79]. A linear mixture model is used to evaluate the performance of the method. The dataset with 64 patient data was used to evaluate the performance.	Sahlgrenska University Hospital, Gothenburg, Sweden	This model has considerable performance in the analysis.	The model has a lower efficiency in analyzing the nonlinear relation in the features.
Convolutional neural network (CNN) model is applied for the segmentation of SAH [80]. Voxel-wise segmentation was used for the segmentation. This model is evaluated on two datasets, and performance is analyzed.	Collaborative European neurotrauma effectiveness research in TBI study	The CNN has the higher efficiency in the segmentation. The model has the higher performance in the analysis.	The CNN model convolution and pooling process create more data for the training, and this creates an overfitting problem. The model has an overfitting problem that affects the performance of the model.
A multilevel linear regression model is applied for the relational analysis of heart rate variability (HRV) and SAH [81]. EEG data of SAH patients were collected to evaluate the performance of the model.	Columbia University Medical Center Institutional Review Board	The model has a higher performance in the feature analysis.	Relevant features were required to be extracted to analyze the HRV, and effective classifier is required to analyze the relation between HRV and SAH.
The elastic net logistic regression model is applied for the prediction of SAH [82]. EEG and clinical factors data were used for the prediction. This model is evaluated in a large dataset to analyze the performance.	Nonelective cEEG at Yale University/Yale New Haven Hospital, Brigham and Women's Hospital, or Emory University Hospital	The model has considerable performance in the prediction. This method effectively analyses the EEG data.	The feature relations in EEG and clinical factors are not effectively analyzed.
Random forest with conditional inferences trees were optimized to predict the SAH [83]. The feature importance is analyzed in this model. The dataset of 630 SAH patients was used to evaluate the performance of the model.	World Federation of Neurosurgical Societies (WFNS)	The random forest-based model has considerable performance in the dataset. The feature importance helps to improve efficiency.	The random forest model is ineffective when a number of trees is more and has overfitting when a number of trees is less.
The faster recurrent convolution neural network (RCNN) model is applied for cerebral aneurysm detection in CT images [84]. The collected dataset is used to evaluate the performance of the model.	Dataset collected from three medical centers.	The deep learning method has a higher performance in detection.	The faster RCNN model generates more data instance to train the network that creates an overfitting problem. Overfitting problem affects the performance of the model. The parameter selection process requires for optimal performance of a network.
Logistic regression model for prediction of SAH and evaluated based on Glasgow Outcome Scale (GOS) [85]. The collected SAH patient dataset was used to evaluate the performance.	Massachusetts General Hospital aSAH database	The evaluation shows that model has the considerable performance. The model has higher efficiency in the feature analysis.	The nonlinear relation between the features of SAH is required for analysis for effective performance. The model has lower efficiency in feature relation analysis.
Method: a multivariate logistic regression model Dataset: in-hospital Mortality in patients with sub arachnoid hemorrhage [86]. Variables relating to their demographic characteristics (age and sex), comorbidities (assessed by Charlson index), SAH (delayed hospital arrival and symptomatology at onset), and severity	Dataset collected from the University Hospital Complex of A Coruña (Spain).	A multivariate logistic regression model was developed to predict the likelihood of in-hospital mortality, adjusting it exclusively for variables present on admission. A predictive equation of in-hospital mortality was then computed based on model's coefficients, along with a point-based risk-scoring system.	Although a multicollinearity analysis was performed, it cannot be ruled out that this issue could have influenced the associated effect sizes and maybe the associations themselves. Finally, this study only represents the clinical experience at our hospital, and so, our results must be validated externally with an independent cohort.
The acute infarction area of diffusion-weighted imaging (DWI) and hypoperfusion of perfusion-weighted imaging (PWI) was labeled manually. Two forms of datasets (volume of interest [VOI] data sets and slice data sets) were analyzed, respectively [87].	Nanjing First Hospital and the Affiliated Jiangning Hospital of Nanjing Medical University	The developed DMTC model in an independent external validation set, and comparing it with the training set, both the VOI data set and the slice data set had good performance in predicting HT, which showed good generalization ability.	First, the sample size is relatively small. Finally, as a result of the sample size, patients receiving bridging therapy were also enrolled, Health Quality Ontario demonstrated that EVT did not show an increased incidence of clinically relevant HT in comparison with IVT.
Multilayer perceptron (MLP), Naïve Bayes, and SVM methods were applied for the prediction process [88].	CT scan images of Charité Universitaetsmedizin Berlin were used to test the performance.	The developed method has considerable performance in prediction process.	The developed model has the imbalance data problem.
Logistic regression model is applied for the prediction process [89].	Teaching hospital in Barcelona (Spain)	The developed method has considerable performance in the risk factor analysis.	The developed method has lower performance in assumption of linearity between dependent and independent variables.

RETRACTED

## Data Availability

No data were used to support this study.
